# Laparoscopic Radical Hysterectomy Combined with Neoadjuvant Chemotherapy for Cervical Cancer Patients Effectively Improves Immune Function

This article has been retracted.

**DOI:** 10.1155/2022/3611174

**Published:** 2022-09-14

**Authors:** Mo Liu, Hongping Wang, Shengye Du, Wenying Li, Fei Xuan, Yinghui Zhao, Na Li

**Affiliations:** ^1^Department of Gynecology and Obstetrics, People's Hospital Affiliated to Shandong First Medical University, Jinan 271199, Shandong Province, China; ^2^Department of Oncology, People's Hospital Affiliated to Shandong First Medical University, Jinan 271199, Shandong Province, China; ^3^Department of Chinese Medicine Gynecology, People's Hospital Affiliated to Shandong First Medical University, Jinan 271199, Shandong Province, China

## Abstract

**Objective:**

To evaluate the clinical efficacy of neoadjuvant chemotherapy plus laparoscopic radical hysterectomy for cervical cancer and the effect on the immune function of patients.

**Methods:**

Between January 2021 and December 2021, 42 patients with cervical cancer diagnosed and treated at our hospital were recruited and randomly assigned at a 1 : 1 ratio to receive neoadjuvant chemotherapy plus open radical hysterectomy (control group) or neoadjuvant chemotherapy plus laparoscopic radical hysterectomy (treatment group) (study group). Outcome measures included surgical indices, clinical outcomes, and immunological function.

**Results:**

There were no significant differences in the operative time between the two groups (*P* > 0.05). Patients receiving laparoscopic surgery had significantly less intraoperative bleeding and shorter time lapse before postoperative anal exhaustion, time lapse before out-of-bed activities, and hospital stay versus patients receiving open surgery (*P* < 0.05). Laparoscopic surgery resulted in a significantly higher efficacy (90.48%) versus open surgery (57.14%) (*P* < 0.05). After treatment, patients in the study group showed lower levels of carcinoembryonic antigen (CEA), squamous cell carcinoma antigen (SCC-Ag), and cancer antigen (CA125) than those in the control group (*P* < 0.05). After treatment, patients given laparoscopic surgery showed significantly lower CD^3+^, CD^4+^, and CD^8+^ levels and higher CD^4+^/CD^8+^ levels versus those with open surgery (*P* < 0.05). The postoperative conditions of the two groups, including recatheterization, postoperative blood transfusion, and secondary anti-inflammation were not significantly different (*P* > 0.05). The study group showed a significantly lower incidence of complications (19.05%) than the control group (71.43%) (*P* < 0.05). Patients in the study group had a lower reoperation rate and a higher survival rate (0.00%, 95.24%) than those in the control group (19.05%, 66.67%) (*P* < 0.05).

**Conclusion:**

Neoadjuvant chemotherapy plus laparoscopic radical hysterectomy effectively improves clinical efficacy, lowers cancer marker levels, improves patients' immune function, reduces the risk of adverse events, and improves patients' prognosis with less intraoperative bleeding, less trauma, faster postoperative recovery, and shorter hospital stay for cervical cancer patients.

## 1. Introduction

Human papillomavirus (HPV) is a high-risk factor for cervical cancer [1], and about 10% of women suffering HPV infection on their cervix develop long-lasting HPV infections, resulting in a high risk for cervical cancer [2]. According to 2018 World Health Organization (WHO) statistics, there were about 569,000 new cases of cervical cancer worldwide, with an incidence of 13/100,000 and a mortality rate of 7/100,000, 84% of which were found in economically underdeveloped countries [3, 4]. Early-stage cervical cancer is mostly asymptomatic [5], while disease progression may result in vaginal bleeding and vaginal drainage [6, 7]. Most cervical cancer cases are aged 40-50 years, but its incidence in the young population has also been increasing in recent years [8]. The incidence of cervical cancer is strongly associated with the level of development, with incidence rates at least four times higher in countries with low Human Development Index (HDI) rankings. Projections of cervical cancer incidence in 2030, estimated on the basis of demographic factors, suggest a 2% increase in the global burden of cervical cancer, which is balanced with the current rate of decline [9].

Molecularly targeted therapies offer a new perspective for the precise treatment of cancer patients. Molecularly targeted drugs are characterized by high specificity and low side effects and have a broad application prospect in the treatment of cancer. Among the molecularly targeted drugs for cervical cancer, the VEGF inhibitor bevacizumab is used for patients with recurrent and metastatic cervical cancer [10], which inhibits the growth and metastasis of cervical cancer by blocking neovascularization. Currently, the prosperous development of bioinformatics provides various new ideas, such as rRNA, miRNA, and lncRNA prediction models to provide certain insights into cancer treatment and drug design. At present, surgery is the main treatment for early-stage cervical cancer, while radiotherapy is administered to patients with mid- to late-stage cervical cancer and those who are intolerant to surgery. Chemotherapy is an important adjuvant therapy for cervical cancer treatment that eliminates microscopic lesions and improves the survival rate of patients. With the advancement of science and technology, advanced technologies such as imaging technology, computer technology, and molecular biotechnology have greatly enhanced the diagnosis and treatment of cervical cancer [11].

Surgery combined with preoperative neoadjuvant chemotherapy (intravenous or arterial infusion chemotherapy) is clinically employed to reduce tumor lesions and control subclinical metastases [12, 13], and the commonly used chemotherapeutic agents include cisplatin, carboplatin, paclitaxel, bleomycin, ifosfamide, and fluorouracil [13]. Traditional open radical hysterectomy for cervical cancer includes extensive hysterectomy, bilateral adnexal resection, and pelvic lymph node dissection [14]. Less trauma, less pain, avoidance of injury to abdominal wall muscles, blood vessels, and similar nerves, fewer postoperative complications, less wound infection, and prevention of abdominal irritation and contamination caused by exposure to dust and bacteria in the air are all advantages of laparoscopic radical hysterectomy for cervical cancer. [15].

The present study was conducted to evaluate the clinical efficacy of neoadjuvant chemotherapy plus laparoscopic radical hysterectomy for cervical cancer and the effect on the immune function of patients, so as to provide data and reference for subsequent studies.

## 2. Materials and Methods

### 2.1. Participants

Between January 2021 and December 2021, 42 patients with cervical cancer (aged 28-65 years, mean age of 43.98 ± 7.2 years) diagnosed and treated in our hospital were recruited and assigned via the random method (June 2021 as the cut-off point) to receive neoadjuvant chemotherapy plus open radical hysterectomy (control group, *n* = 21) or neoadjuvant chemotherapy plus laparoscopic radical hysterectomy (study group, *n* = 21).

The randomization was carried out using an online web-based randomization tool (freely available at http://www.randomizer.org/). For concealment of allocation, the randomization procedure and assignment were managed by an independent research assistant who was not involved in the screening or evaluation of the participants.

We estimated that with a sample size of 21 patients assigned to receive study group treatment and 21 assigned to receive control group treatment, the study would have more than 99% power to detect a between-group difference in the relevant indicators for this study.

The trial was done in accordance with the standards of Good Clinical Practice and the Declaration of Helsinki. The trial protocol and all amendments were approved by the appropriate ethics body at each participating institution. All patients provided written informed consent before enrolment. The trial protocol has been published online and is available with the full text of this article. Ethics number: NU-UI20210102.

### 2.2. Inclusion and Exclusion Criteria

Inclusion criteria: patients who met the diagnostic criteria related to cervical cancer in the Chinese Common Malignant Tumor Diagnostic and Treatment Standard [16]; with an expected survival of >3 months; with consciousness and normal communication ability; aged 20 years old and above; with WHO standard physical index ≤2; without previous treatment; with normal complete blood cytology, cardiopulmonary function, liver and kidney function, electrocardiogram, and chest radiograph; who provided written informed consent were included.

Exclusion criteria: patients with serious heart, brain, and other dysfunction and immune system diseases; with abnormal coagulation function or hematological system diseases; with contraindications to treatment related to this study; with severe systemic or uncontrolled disease (e.g., infection, central nervous system disease, and metabolic disease) that interferes with the use of chemotherapeutic agents; who were pregnant or breastfeeding; with other malignancies; with psychiatric disorders; with neurological disorders; or with incomplete clinical data were excluded.

### 2.3. Treatment

All patients underwent routine examinations before chemotherapy, including blood routine testing, coagulation function testing, liver and kidney function testing, electrocardiogram, and chest X-ray.

Patients in the control group received neoadjuvant chemotherapy plus an open hysterectomy. Patients received 1.5 mg of dexamethasone tablets (Approval No. H44024618, Guangdong Nanguo Pharmaceutical Co., Ltd.) orally 12 h and 6 h before chemotherapy. Then, the patients received 50 mg of diphenhydramine hydrochloride injection (State Drug Quantifier H37020713, Shandong Xinhua Pharmaceutical Co.) through intramuscular injection for 0.5 h, 300 mg of cimetidine injection (GMPZ H37023309, Shandong Dongfangming Pharmaceutical Group Co.) through intravenous injection, 10 mg of dexamethasone sodium phosphate injection (Guopharm Quantifiers H41020035, Sinopharm Group Rongsheng Pharmaceutical Co.) through intravenous injection, and 135 mg/m^2^ of paclitaxel injection (State Drug Quantifier H20067186, Biomedical Engineering Center of Hebei Medical University) and 60 mg/m^2^ of cisplatin injection (State Drug Quantifier H37021358, Qilu Pharmaceutical Co.) through intravenous injection within 3 h. An identical neoadjuvant chemotherapy regimen was introduced to the patients in the study group.

The surgery was performed 3-7 days after the menstruation period. After general anesthesia, an extensive hysterectomy and pelvic lymph node dissection were performed after opening the abdomen layer by layer through a midline or left longitudinal incision for inspection of the pelvic and abdominal cavities.

The patients in the study group received neoadjuvant chemotherapy plus laparoscopic radical hysterectomy. The laparoscopic radical hysterectomy was performed 3-7 days after the menstruation period. Oral antibiotics were administered 3 days before surgery, vaginal irrigation was performed 2-3 days before surgery, and a cleansing enema was administered 1 day before surgery. After anesthesia, the uterus was suspended with bilateral coracoid sutures, and the abdominal wall was stretched bilaterally to elevate the uterus. A 10 mm trocar was placed at the inferior border of the umbilicus followed by the placement of the laparoscope and the establishment of a CO_2_ pneumoperitoneum with a pressure of 13-14 mmHg. A 5 mm trocar was placed at McBurney's point in the right lower abdomen and at 1 cm medial to the left anterior superior iliac spine, and a 5 mm or 10 mm trocar was placed at an equidistant point in the umbilicus as an operating port for inspection of the pelvic and abdominal cavities. The right lateral pelvic peritoneum was opened and the outer 1/3 of the right round ligament was severed by ultrasonic knife, the left round ligament was treated in the same way, and the proximal end of the right round ligament and its attachments were lifted to stretch the pelvic funnel ligament. The peritoneum above was severed, the posterior lobe of the broad ligament was separated, the ovarian artery was revealed, the vessels were closed bipolarly, and the ovarian artery was severed with an ultrasonic knife. The proximal end of the round ligament was lifted, the anterior lobe of the broad ligament was cut along the parametrium, the peritoneum was separated, the bladder-uterine reflex peritoneum was cut transversely, and the bladder was pushed down to the level of the external cervical os. The posterior peritoneum was incised at the severed end of the funnel ligament of the pelvis toward the ipsilateral common iliac artery. The anterior and posterior lobes of the broad ligament were cut transversely at the inferior border of the right funnel ligament, then the anterior and posterior peritoneum were cut downward, respectively, and the bladder was pushed down in the same way as the left side. The ultrasonic knife was used to sever the ligamentous ligament of the right ovary. The fatty connective tissue over the psoas major muscle was separated to reveal the genitofemoral nerve. The lymphoid adipose tissue in front of and around the right common and external iliac arteries was removed from above and below. The lymphatic adipose tissue in front of the external iliac vein was freed and pulled outward to reveal the internal iliac artery, and the lymphatic adipose tissue between them was separated. The deep inguinal lymph nodes were separated at the lowermost end of the iliac vessels, distal to the intersection of the spinocranial veins. The bladder was lifted medially to expose the external iliac vein to isolate the foramen ovale nerve. The lymphatic adipose tissue of the foramen ovale was separated from the bottom up above the foramen ovale nerve, and the left pelvic lymph nodes were cleansed in the same way. The loose connective tissue between the vaginal posterior wall and the rectum anterior wall was detached. The bladder was pulled down after the anterior lobe of the wide ligament and the peritoneal retrusion of the bladder were opened. The ureter was totally moved aside after bipolar electrocoagulation was used to detach the anterior and posterior lobes of the ureteral tube bilaterally. The utero-rectal gap was expanded and the rectum pushed downward. The bilateral uterosacral ligaments were dissected by bipolar electrocoagulation 3 cm from the parametrium. The adjacent tissues of both main ligaments were dissected by bipolar electrocoagulation 3 cm from the parametrium after blocking the blood flow using a bipolar or ultrasonic knife. The anterior and posterior domes were cut open and the uterus was excised. The vaginal stump was sutured, the abdominal cavity was irrigated to examine for active bleeding, drainage was performed, and the instruments were removed.

### 2.4. Outcome Measures

1. *Surgical Indices*. The surgical indices of the two groups were recorded, including the operation time, intraoperative bleeding, time lapse before postoperative anal exhaustion, time lapse before out-of-bed activity, and hospital stay
2. *Clinical Efficacy*. With reference to WHO efficacy criteria, ultrasound results, and MRI results, the efficacy was evaluated and divided into four levels: complete remission (CR), partial remission (PR), stable disease (SD), and progressive disease (PD). CR: tumor disappeared visually, and no new lesions occurred. PR: tumor volume reduced by >50% and no new lesions occurred. SD: tumor volume reduced by <50%. PD: tumor volume did not reduce, or new lesions occurred. Total clinical efficiency = (CR + PR)/total number of cases x 100%.
3. *Tumor Markers*. 2-3 mL of morning fasting venous blood was collected from all patients before and after treatment and centrifugated at 3500 r/min to isolate the serum which was stored at −70°C for assays. The levels of serum carcinoembryonic antigen (CEA), squamous cell carcinoma antigen (SCC-Ag), and cancer antigen (CA125) were determined using an automatic electrochemiluminescence immunoassay analyzer
4. *Immune Function Indices*. 2-3 mL of morning fasting venous blood was collected from all patients before and after treatment, and the serum was separated by centrifugation at 3500 r/min and stored at −70°C for assays. Flow cytometry was used to determine the CD^3+^, CD^4+^, and CD^8+^ levels in the two groups, and CD^4+^/CD^8+^ was calculated
5. *Postoperative Conditions*. The postoperative conditions of patients in both groups were recorded in detail, including recatheterization, postoperative blood transfusion, and secondary anti-inflammation
6. *Complications*. The occurrence of complications, including intestinal obstruction, urinary tract infection, lymphatic cyst, pelvic-abdominal infection, and wound infection was recorded in detail in both groups
7. *Follow-Up*. The patients were followed up for 21 months by home visit or telephone, and the reoperation and survival of the two groups were recorded in detail for comparison

### 2.5. Statistical Analysis

The mean difference between the two groups was tested using the student *t*-test for normally distributed variables and the Mann–Whitney *U* test for nonnormal variables.

Data analyses were performed using the SPSS22.0. The measurement data are expressed as (mean ± SD) and analyzed using the independent *t*-test, and the count data are expressed as (%) and analyzed using the chi-squared test. Differences were considered statistically significant at *P* < 0.05.

## 3. Results

### 3.1. Patient Characteristics

There were 21 patients in the study group, aged 30-65 years, an average age of 44.21 ± 6.18 years, tumor diameter of 4-9 cm, an average of 5.98 ± 1.11 cm, 14 cases of stage Ib2 and 7 cases of stage IIa in terms of the International Federation of Gynecology and Obstetrics (FIGO) staging, 16 cases of pathological type squamous carcinoma, 3 cases of adenocarcinoma, and 2 cases of adenosquamous carcinoma in terms of pathological type. There were 21 patients in the study group, aged 28-61 years, average age of 43.56 ± 7.88 years, tumor diameter of 4-9 cm, an average of 6.12 ± 1.03 cm, 15 cases of stage Ib2 and 6 cases of stage IIa in terms of the International Federation of Gynecology and Obstetrics (FIGO) staging, 15 cases of pathological type squamous carcinoma, 5 cases of adenocarcinoma, and 1 case of adenosquamous carcinoma in terms of pathological type. There were no significant differences in terms of patient characteristics between the two groups (*P* > 0.05) (Table 1).

### 3.2. Surgical Indices

There were no significant differences in the operative time between the two groups (*P* > 0.05). In comparison to patients who had open surgery, those who underwent laparoscopic surgery had much less intraoperative bleeding and a shorter period before postoperative anal tiredness, time lapse before out-of-bed activities, and hospital stay (*P* < 0.05) (Table 2).

### 3.3. Clinical Efficacy

There were 8 (38.10%) cases of CR, 11 (52.38%) cases of PR, 1 (4.76%) case of SD, and 1 case of PD in the study group, and there were 4 (19.05%) cases of CR, 8 (38.10%) cases of PR, 6 (28.57%) cases of SD, and 3 (14.29%) cases of PD in the control group. Laparoscopic surgery resulted in a significantly higher efficacy (90.48%) versus open surgery (57.14%) (*P* < 0.05) (Table 3).

### 3.4. Tumor Markers

The two groups had similar tumor marker levels before treatment (*P* > 0.05). Patients in the study group had lower levels of CEA, SCC-Ag, and CA125 after therapy than those in the control group (*P* < 0.05) (Table 4).

### 3.5. Immune Function

There were no significant differences in the immune function indices before treatment between the two groups (*P* > 0.05). After treatment, patients given laparoscopic surgery showed significantly lower CD^3+^, CD^4+^, and CD^8+^ levels and higher CD^4+^/CD^8+^ levels versus those given open surgery (*P* < 0.05). (Table 5).

### 3.6. Postoperative Conditions

The postoperative conditions of the two groups, including recatheterization, postoperative blood transfusion, and secondary anti-inflammation were not significantly different (*P* > 0.05) (Table 6).

### 3.7. Complications

There were 1 (4.76%) case of intestinal obstruction, 2 (9.52%) cases of urinary tract infection, and 1 (4.76%) case of lymphatic cyst in the study group, and 1 (4.76%) case of intestinal obstruction, 6 (28.57%) cases of urinary tract infection, 4 (19.05%) cases of lymphatic cyst, 2 (9.52%) cases of pelvic abdominal infection, and 2 (9.52%) cases of wound infection in the control group. The study group showed a significantly lower incidence of complications (19.05%) than the control group (71.43%) (*P* < 0.05) (Table 7).

### 3.8. Follow-Up

Patients in the study group had a lower reoperation rate and a higher survival rate (0.00%, 95.24%) than those in the control group (19.05%, 66.67%) (*P* < 0.05) (Table 8).

## 4. Discussion

Cervical cancer has the fourth highest incidence and mortality rate of all cancers. A global survey of the status of 36 malignant tumors in 185 countries reported that cervical cancer had about 570,000 new cases in 2018, accounting for 6.6% of new cases of malignant tumors in women, and as many as 310,000 deaths (7.5%). In China, the number of cervical cancer cases reached 111,000 and 34,000 deaths in 2015, and the incidence has shown an increasing trend [17, 18]. At present, early-stage cervical cancer is mostly managed by surgery, but still, 30% of patients fail to obtain favorable clinical results, with poor clinical prognosis and postoperative recurrence rates of up to 10-20%, mainly related to factors such as the International Federation of Gynecology and Obstetrics (FIGO) staging, choroidal cancer embolism, pelvic lymph node metastasis, and the specificity of its surrounding tissues. Thus, postoperative cervical cancer with adjuvant radiotherapy for comprehensive intervention to control postoperative recurrence has become a highly desired treatment modality for early-stage cervical cancer [19, 20].

Neoadjuvant chemotherapy is administered to patients for 2-3 cycles followed by a subsequent treatment plan [21]. Laparoscopic radical hysterectomy for cervical cancer features less trauma, mild pain, fewer postoperative complications such as abdominal wall weakness and abdominal wall incisional hernia, and a lower risk of infection than traditional open incision [22]. The theoretical basis of neoadjuvant chemotherapy for cervical cancer is as follows: (1) the local vascular bed of the tumor site is relatively intact before radiation therapy or surgery for patients, which allows for good performance of chemotherapeutic drugs; (2) it significantly reduces the proportion of hypoxic cells in tumor tissues and increases the sensitivity to radiation therapy; (3) it reduces tumor volume, improves local infiltration and parametrial tumors, and lowers the possibility of tumor spread during surgery; (4) before preoperative or pelvic radiotherapy, patients are generally in better condition with high tolerance of chemotherapy, which significantly reduces the toxicity of chemotherapeutic drugs; (5) it provides favorable conditions for management of subclinical lesions, thus reducing the risk of recurrence and metastasis; (6) preoperative chemotherapy provides an objective evaluation of the sensitivity of tumor response to chemotherapy. In neoadjuvant chemotherapy for cervical cancer, cisplatin is the most effective agent and DNA is an important target for cisplatin [23, 24].

In the present study, patients receiving laparoscopic surgery had significantly less intraoperative bleeding and shorter time lapse before postoperative anal exhaustion, time lapse before out-of-bed activities, and hospital stay versus patients receiving open surgery; laparoscopic surgery resulted in a significantly higher efficacy (90.48%) versus open surgery (57.14%). The reason may be that neoadjuvant chemotherapy treatment obviously reduces the tumor volume, and radical laparoscopic hysterectomy for cervical cancer results in small surgical wounds, less intraoperative bleeding and surgical damage, a clear surgical vision, and high safety. Furthermore, it maximizes the complete resection of the tumor and reduces the risk of disease recurrence and metastasis, and chemotherapy decreases the viability of tumor cells and facilitates postoperative recovery, demonstrating that preoperative neoadjuvant chemotherapy lowers the difficulty of surgery by preoperatively shrinking the tumor volume, and its combination with laparoscopic radical cervical cancer surgery provides expanded suture options.

It has been suggested [25] that cervical cancer is associated with severe damage to the cellular immune function of the body. Alterations in the levels of CD^3+^, CD^4+^, and CD^8+^ are indicative of the immune status of the body, and serum CEA, SCC-Ag, and CA125 are tumor molecular markers closely related to cervical cancer with high detection sensitivity. The results of the present study showed that the differences in tumor markers and immune function levels between the two groups before treatment were not statistically significant. After treatment, the study group showed significantly lower levels of CEA, SCC-Ag, CA125, CD^3+^, CD^4+^, and CD^8+^ and a higher CD^4+^/CD^8+^ level than the control group. The main component of paclitaxel is the natural anticancer drug paclitaxel, which provides effective antitumor effect and has obvious effect on uterine cancer and breast cancer. Through preoperative neoadjuvant chemotherapy, cisplatin combined with paclitaxel further inhibits tumor cell proliferation, reduces tumor cell growth, shrinks tumor volume, decreases tumor cell viability, reduces intraoperative spread, lowers surgical difficulty, and promotes postoperative recovery. In addition, neoadjuvant chemotherapy has a strong tumor-killing effect, which reduces tumor load and thus tumor-induced immunosuppression. The denaturation of tumor proteins after chemotherapy treatment induces the formation of other antigens of the same type, which in turn increases the immune function of the body [26, 27].

Studies have found that neoadjuvant chemotherapy provides prominent benefits in the treatment of cancer. Paclitaxel is a new intracellular microtubule drug that binds to tubule beta sites specifically in vivo, effectively preventing microtubule protein breakdown and limiting cell proliferation and release. Platinum medicines inhibit DNA repair enzymes, reduce tumor volume, increase blood circulation in tumor tissues, and efficiently boost chemotherapeutic drug penetration into tumor tissues [28]. Herein, neoadjuvant chemotherapy plus laparoscopic radical cervical cancer treatment completely removes cervical cancer lesions, significantly lowers the levels of molecular tumor markers and tumor metastasis-related factors in cervical cancer patients, and corrects the immune dysfunction, which is consistent with the results of previous research [29]. Furthermore, the study group showed a significantly lower incidence of complications, lower reoperation rate, and a higher survival rate than the control group, indicating that neoadjuvant chemotherapy plus laparoscopic radical hysterectomy is associated with a better prognosis versus open surgery [30]. Traditional open surgery includes large surgical incisions and significant damage to the abdominal wall muscles, blood vessels, and related nerves, resulting in postoperative complications, compromised prognosis, and a high risk of reoperation. Laparoscopic radical cervical cancer surgery is a minimally invasive method that eliminates the stimulation and contamination of the abdominal cavity by airborne microorganisms, resulting in few postoperative problems, excellent safety, and a favorable patient prognosis [31]. In addition, the absence of significant differences in terms of postoperative conditions of the two groups of patients, including recatheterization, postoperative blood transfusion, and secondary anti-inflammation, may be attributed to the small sample size of the present study [32]. Therefore, subsequent multiple center studies with a larger sample size will be conducted to provide more reliable data.

Neoadjuvant chemotherapy before radical surgery for cervical cancer significantly reduces the tumor diameter and effectively inhibits the proliferation of tumor cells, which shrinks the tumor size and improves the patient's prognosis. In addition, neoadjuvant chemotherapy also allows for a reduction in tumor extent and prevents complications due to excessive surgical extent, such as rectal injury and bladder injury. This study has the following limitations: (1) the sample size of this study was small; (2) the follow-up of patients was relatively short; (3) animal experiments in vivo and ex vivo have not been conducted in this study, and the mechanism of the treatment modality of this study has not been investigated.

## 5. Conclusion

Neoadjuvant chemotherapy plus laparoscopic radical hysterectomy for cervical cancer patients effectively improves clinical efficacy, lowers cancer marker levels, enhances patients' immune function, reduces the risk of adverse events, and improves patients' prognosis with less intraoperative bleeding, less trauma, faster postoperative recovery, and shorter hospital stay.

## Figures and Tables

**Table 1:** Patient characteristics ($\bar{\text{x}}\pm \text{s}$).

Group	*n*	Age		Tumor diameter		FIGO staging		Pathological type		
		Range	Mean	Range	Mean	Ib2	IIa	Squamous carcinoma	Adenocarcinoma	Adenosquamous carcinoma
Study	21	30-65	44.21 ± 6.18	4-9	5.98 ± 1.11	14	7	16	3	2
Control	21	28-61	43.56 ± 7.88	4-9	6.12 ± 1.03	15	6	15	5	1
*t*	—	—	0.297	—	0.424	—	—	—	—	—
*P* value	—	—	0.768	—	0.674	—	—	—	—	—

Note: FIGO: the International Federation of Gynecology and Obstetrics.

**Table 2:** Surgical indices ($\bar{\text{x}}\pm \text{s}$).

Group	*n*	Operation time (min)	Intraoperative bleeding (ml)	Time-lapse before postoperative anal exhaustion (*d*)	Time-lapse before out-of-bed activities (*d*)	Hospital stay (*d*)
Study	21	185.23 ± 15.92	150.84 ± 98.48	1.72 ± 0.52	2.08 ± 0.82	7.09 ± 1.08
Control	21	191.17 ± 18.37	893.15 ± 225.54	2.93 ± 0.98	3.97 ± 1.02	12.31 ± 2.31
*t*	—	1.120	13.822	4.998	6.618	9.381
*P* value	—	0.269	<0.001	<0.001	<0.001	<0.001

**Table 3:** Clinical efficacy (%).

Group	*n*	CR	PR	SD	PD	Total efficacy
Study	21	8 (38.10)	11 (52.38)	1 (4.76)	1 (4.76)	19 (90.48)
Control	21	4 (19.05)	8 (38.10)	6 (28.57)	3 (14.29)	12 (57.14)
*x* ^2^	—	6.035				
*P* value	—	0.014				

Note: CR is complete remission; PR is partial remission; SD is stable disease; PD is progressive disease.

**Table 4:** Tumor marker levels ($\bar{\text{x}}\pm \text{s}$).

Group	*n*	CEA(ng/L)		SCC-ag(*μ*g/mL)		CA125(*μ*g/L)	
		Before treatment	After treatment	Before treatment	After treatment	Before treatment	After treatment
Study	21	44.28 ± 3.48	29.98 ± 3.55^∗^	1.25 ± 0.37	0.97 ± 0.23^∗^	65.17 ± 3.34	47.17 ± 2.18^∗^
Control	21	44.35 ± 3.17	32.95 ± 4.08^∗^	1.26 ± 0.41	1.21 ± 0.22^∗^	65.25 ± 3.17	51.34 ± 2.91^∗^
*t*	—	0.068	2.517	0.083	3.456	0.008	5.256
*P* value	—	0.946	0.016	0.934	0.001	0.937	<0.001

Note: ∗ indicates a significant difference (*P* < 0.05) between pre- and posttreatment comparisons in the same group. CEA is serum carcinoembryonic antigen; SCC-Ag is squamous cell carcinoma antigen; CA125 is cancer antigen 125.

**Table 5:** Immune function indices levels ($\bar{\text{x}}\pm \text{s}$).

	Timepoints	Study (*n* = 21)	Control (*n* = 21)	*t*	*P* value
CD^3+^(%)	Before treatment	50.12 ± 2.51	50.17 ± 2.44	0.065	0.948
	After treatment	41.15 ± 1.91^∗^	45.87 ± 1.88^∗^	8.071	<0.001

CD^4+^(%)	Before treatment	35.12 ± 1.27	35.34 ± 1.28	0.559	0.579
	After treatment	31.17 ± 1.08^∗^	34.08 ± 1.33^∗^	7.784	<0.001

CD^8+^(%)	Before treatment	35.65 ± 1.31	35.88 ± 1.56	0.517	0.608
	After treatment	30.29 ± 1.23^∗^	33.95 ± 1.27^∗^	9.487	<0.001

CD^4+^/CD^8+^	Before treatment	1.00 ± 0.03	1.00 ± 0.04	0.000	1.000
	After treatment	1.05 ± 0.06^∗^	1.01 ± 0.03^∗^	2.733	0.009

Note: ∗ indicates a significant difference (*P* < 0.05) between pre- and post-treatment comparisons in the same group.

**Table 6:** Postoperative conditions (%).

Group	*n*	Recatheterization	Postoperative blood transfusion	Anti-inflammation
Study	21	3 (14.29)	1 (4.76)	6 (28.57)
Control	21	4 (19.05)	2 (9.52)	7 (33.33)
*x* ^2^	—	0.171	0.359	0.111
*P* value	—	0.679	0.549	0.739

**Table 7:** Complications (%).

Group	*n*	Intestinal obstruction	Urinary tract infection	Lymphatic cyst	Pelvic abdominal infection	Wound infection	Total incidence
Study	21	1 (4.76)	2 (9.52)	1 (4.76)	0 (0.00)	0 (0.00)	4 (19.05)
Control	21	1 (4.76)	6 (28.57)	4 (19.05)	2 (9.52)	2 (9.52)	15 (71.43)
*x* ^2^	—	11.629					
*P* value	—	0.001					

**Table 8:** Follow-up (%).

Group	*n*	Reoperation rate	Survival rate
Study	21	0 (0.00)	20 (95.24)
Control	21	4 (19.05)	14 (66.67)
*x* ^2^	—	4.421	5.559
*P* value	—	0.035	0.018

## Data Availability

All data generated or analysed during this study are included in this published article.
